The article "PDHA1 gene knockout in prostate cancer cells results in metabolic reprogramming towards greater glutamine dependence" was retracted in 2025. Reasons: manipulated images; an official misconduct investigation; duplicated images; overlap with earlier publications.

# *PDHA1* gene knockout in prostate cancer cells results in metabolic reprogramming towards greater glutamine dependence

**DOI:** 10.18632/oncotarget.10782

**Published:** 2016-07-22

**Authors:** Yaqing Li, Xiaoran Li, Xiaoli Li, Yali Zhong, Yasai Ji, Dandan Yu, Mingzhi Zhang, Jian-Guo Wen, Hongquan Zhang, Mariusz Adam Goscinski, Jahn M. Nesland, Zhenhe Suo

**Affiliations:** ^1^ Department of Oncology, The First Affiliated Hospital of Zhengzhou University, Zhengzhou, Henan Province, China; ^2^ Department of Pathology, The Norwegian Radium Hospital, Oslo University Hospital, University of Oslo, Montebello, Oslo, Norway; ^3^ Department of Pathology, The Institute of Clinical Medicine, Faculty of Medicine, University of Oslo, Montebello, Oslo, Norway; ^4^ Institute of Clinical Medicine, The First Affiliated Hospital of Zhengzhou University, Zhengzhou, Henan Province, China; ^5^ Department of Anatomy, Histology and Embryology, Peking University Health Science Center, Peking University, Beijing, China; ^6^ Department of Surgery, the Norwegian Radium Hospital, Oslo University Hospital, University of Oslo, Oslo, Norway

**Keywords:** PDHA1 gene knockout, metabolic reprogramming, glutamine dependence, prognosis, GC-MS analysis

## Abstract

Alternative pathways of metabolism endowed cancer cells with metabolic stress. Inhibiting the related compensatory pathways might achieve synergistic anticancer results. This study demonstrated that pyruvate dehydrogenase E1α gene knockout *(PDHA1* KO) resulted in alterations in tumor cell metabolism by rendering the cells with increased expression of glutaminase1 (GLS1) and glutamate dehydrogenase1 (GLUD1), leading to an increase in glutamine-dependent cell survival. Deprivation of glutamine induced cell growth inhibition, increased reactive oxygen species and decreased ATP production. Pharmacological blockade of the glutaminolysis pathway resulted in massive tumor cells apoptosis and dysfunction of ROS scavenge in the LNCaP *PDHA1* KO cells. Further examination of the key glutaminolysis enzymes in human prostate cancer samples also revealed that higher levels of GLS1 and GLUD1 expression were significantly associated with aggressive clinicopathological features and poor clinical outcome. These insights supply evidence that glutaminolysis plays a compensatory role for cell survival upon alternative energy metabolism and targeting the glutamine anaplerosis of energy metabolism via GLS1 and GLUD1 in cancer cells may offer a potential novel therapeutic strategy.

## INTRODUCTION

Cell survival and growth require metabolic pathways that provide energy, precursors and substrates for macromolecular synthesis and other essential functions [1]. Cancer cells have unique metabolic characteristics such as elevated energetic and biosynthetic demands for rapid cell growth and proliferation. The most well known one is the Warburg effect, in which cancer cells consume large amounts of glucose through the glycolysis pathway to produce ATP and lactate even when the oxygen exists [2, 3].

The article "PDHA1 gene knockout in prostate cancer cells results in metabolic reprogramming towards greater glutamine dependence" was retracted in 2025. Reasons: manipulated images; an official misconduct investigation; duplicated images; overlap with earlier publications.

Although cancer cells exhibit high rates of glycolysis, their mitochondrial oxidative phosphorylation (OXPHOS) may remain relatively active and become extensively more reliable on glutamine metabolism since glutamine also represents a major source of carbon molecules that sustain tumor growth-facilitated metabolic pathways. Consequently, cancer cells may become “addicted” to glutaminolysis [4].

The pyruvate dehydrogenase(PDH) functions as a gatekeeper in glucose metabolism by oxidatively decarboxylating pyruvate which generates from glycolysis or other pathways to produce acetyl-CoA for the TCA cycle and separates pyruvate between aerobic and anaerobic metabolisms [5]. Pyruvate decarboxylation catalyzed by pyruvate dehydrogenase E1(PDHA1) is considered to be the rate-limiting step. E1 is composed of two α and two β subunits and the E1α subunit is encodedby the *PDHA1* gene [6, 7]. It has reported that cancer cells frequently exhibit increased expression of the PDH kinase PDK1, which phosphorylates and inactivates PDH [8].

In standard culture, many cancer cells utilize the TCA cycle in which most of the acetyl-CoA is produced from the glucose-derived pyruvate via PDH and most of the anaplerosis is supplied by glutamine [9]. It is known that the glucose-independent glutamine metabolism via TCA cycling maintains the proliferation and survival in human Burkitt lymphoma model P493 [10]. Another report shows that the glutamine oxidation participates in maintaining the TCA cycle and cell survival during impaired mitochondrial pyruvate transport in SFxL glioma cells [11]. The above reports highlight the compensatory ability of glutamine in TCA cycle through glutaminolysis when OXPHOS is defect in cancer cells.

The gatekeeper enzyme of glutaminolysis is glutaminase (GLS), which catalyses the hydrolysis of glutamine to glutamate, the first step of glutaminolysis. Two genes encode GLSs in human cells: GLS1 (also known as kidney-type GLS), and GLS2 (also known as liver-type GLS). GLS1 is ubiquitously expressed in various tissues [12] and frequently activated and/or overexpressed in various types of cancer [12–14], which is mainly attributable to its GLS activity and role in promoting glutamine metabolism [12–15]. In the second step, glutamate dehydrogenase 1(GLUD1) or transaminases produce α-ketoglutarate (αKG) from glutamate to “feed” the TCA cycle [16]. Expression of GLS1 and GLUD1 are increased in many types of cancers compared to normal tissues and the targeted inhibition of these enzymes have been shown to exert antitumor effect by significantly suppressing cancer cell growth and proliferation [14, 17]. It has been indicated that increasing activity of GLS and increasing glutamine consumption correlate with proliferation, migration and invasion of prostate cancer cells [18]. Another report shows that the glutamine transporter ASCT2 (SLC1A5) is highly expressed in prostate cancer samples and chemical or shRNA-mediated inhibition of ASCT2 function in LNCaP and PC-3 prostate cancer cell lines inhibit glutamine uptake, cell cycle progression, mTORC1 pathway activation and cell growth. Furthermore, shRNA knockdown of ASCT2 in PC-3 cell xenografts significantly inhibit tumour growth and metastasis in an *in vivo* study [19].

The article "PDHA1 gene knockout in prostate cancer cells results in metabolic reprogramming towards greater glutamine dependence" was retracted in 2025. Reasons: manipulated images; an official misconduct investigation; duplicated images; overlap with earlier publications.

Although extensive data have indicated the importance of PDH activity to support cell metabolism and growth in proliferating cells [8, 20], the anaplerosis pathway in *PDHA1* gene knockout prostate cancer cells has not been carefully studied yet. Here we used mass spectrometry-based profiling of the 521 metabolites of 29 metabolic pathways/groups to explore the metabolic reprograming in the LNCaP *PDHA1* KO prostate cancer cell line. The purposes of the current study were to explore how cell glutaminolysis metabolic reprograming was influenced after the TCA cycle gatekeeper gene *PDHA1* was knocked out in the prostate cancer LNCaP cell line, and study the role of the glutamine anaplerosis *in vitro* and *in vivo*.

## RESULTS

### *PDHA1* KO forces cells with glutamine dependent metabolism

To explore the intracellular metabolic shift between the LNCaP parental and *PDHA1* KO prostate cancer cells, we examined the glucose and glutamine metabolism in the two groups. Consistent with the increase in glucose utilization (Figure 1A), *PDHA1* KO cells exhibited an increase in glutamine uptake. The glutamine utilization rate after depletion of *PDHA1* was significantly increased (Figure 1B). We next performed a GC-MS based targeted metabolic analysis to gain more insight into the intracellular metabolic reprogramming induced by the inactivation of *PDHA1* gene. Around 521 metabolite sets were tested using the LECO/Fiehn Metabolomics Library. To refine these analyses, the principal component of variable importance projection (VIP) was obtained. The VIP values exceeding 1.0 were first selected as changed metabolites after the multivariate approaches, the significance of each metabolite in-group discrimination was further measured by the Student's t-test (*P*<0.05). Based on these criteria, 47 significantly changed metabolites were identified due to the *PDHA1* gene knockout (Figure 2A).

The article "PDHA1 gene knockout in prostate cancer cells results in metabolic reprogramming towards greater glutamine dependence" was retracted in 2025. Reasons: manipulated images; an official misconduct investigation; duplicated images; overlap with earlier publications.

**Figure 1:** Results of glucose and glutamine consumption examinations As shown in **A.**, the LNCaP *PDHA1* KO cells consume 5.33mg while the parental cells consume only about 2.13mg glucose after 12hrs culture, which show a significant difference with a *P* value less than 0.001. At 24h culture the LNCaP *PDHA1* KO cells consume 3.51mgwhile the parental cells consume about 7.45mg glucose (*P <0.001*). The data are normalized based on cell number in each experiment. Similarly, **B.** shows the results of glutamine consumption. At 24hrs culture the LNCaP *PDHA1* KO cells consume 3.22μmol while the LNCaP parental cells consume only about 1.52μmol L-glutamine, which show a significant difference with a *P* value less than 0.001. At 48hrs culture the LNCaP *PDHA1* KO cells consume 4.01μmol in the medium while the LNCaP parental cells consume about 1.81μmol L-glutamine (*P*=0.000). The uneven cell numbers caused by different division ratio after 24hrs and 48hrs's cultivation were normalized. ***P<0.001.

**Figure 2:** Steady-state comparative metabolomic profiles and glutamine dependence test **A.** The heat map of the 47 significantly changed metabolites in the two cell lines. The color scale is noted in the upper right corner. Each column represents the metabolomics detection result of a treatment group and each row represents the variable results of a metabolite in different cells. The pathway impact and the fold enrichment of the effect of *PDHA1* KO on the metabolites are shown in **B.** and **C.**, respectively. **D.** After 48hrs's culture in medium without glutamine, apparently more *PDHA1* KO cells are detached from the flask while the parental LNCaP cells are still largely attached. The *PDHA1* KO floating cells are verified as apoptotic (right panel). 2mM glutamine addition in the medium improves the cell attachment while 4mM glutamine almost recovers the cell attachment as compared to the parental LNCaP cells, verifying the glutamine dependence of the *PDHA1* KO cells (left panel). The scale bar is 50μm.

*PDHA1* KO cells possessed a nearly 17.37-fold decrease in cellular metabolite N-Acetyl-L-glutamic acid. At the same time, *PDHA1* KO cells also showed a 4.1-fold and 2.0-fold decrease in cellular L-glutamic acid and glutamic acid, respectively the intermediates of glutamine metabolism, indicating high level of glutamine consumption. Furthermore, there was an interesting and unique pattern in the increased accumulation of metabolites associated with the branched chain amino acids metabolism in the *PDHA1* KO cells including a 2.76-fold and 2.82-fold cellular increases in cellular aspartic acid 1 and aspartic acid 2, respectively, and 3.88-fold and 2.87-fold increases in cellular leucine and cellular L-homoserine 1, respectively (Figure 2A).

The article "PDHA1 gene knockout in prostate cancer cells results in metabolic reprogramming towards greater glutamine dependence" was retracted in 2025. Reasons: manipulated images; an official misconduct investigation; duplicated images; overlap with earlier publications.

In addition, the commercial databases including KEGG (http://www.genome.jp/kegg/) and NIST (http://www.nist.gov/index.html) were utilized to search for the altered metabolites. 20 pathways with high difference between the two groups were defined. The pathway impact and enrichment analyses revealed that the *PDHA1* gene knockout in the LNCaP cell line was linked to glycolysis and other glucose-related pathways including the pentose phosphate shunt, fructose metabolism and upregulated glutamate metabolism (Figure 2B and 2C). However, we discovered in our experiments that apparently more *PDHA1* KO cells detached from the flask as early as after 48hrs in medium without glutamine (Figure 2D, left panel). While the parental LNCaP cells still largely attached on the flask, the *PDHA1* KO cells showed areas of floating cells (Figure 2D, right panel), which were verified as apoptotic, indicating a possibility of glutamine dependence of the *PDHA1* KO cells. To further confirm this, we placed the *PDHA1* KO cells in different media with 0mM, 2mM and 4mM glutamine and explored the influence of glutamine on cell growth. It was verified that the 2mM glutamine addition in the medium could improve the cell attachment while 4mM glutamine could almost recover the cell attachment as compared to the parental LNCaP cells, verifying the glutamine dependence of the *PDHA1* KO cells (Figure 2D, left panel).

### *PDHA1* KO cells are more glutaminolysis dependent

Next, we asked whether the metabolomic changes associated with the depletion of *PDHA1* in prostate cancer cells were associated with the protein expression alterations in corresponding key metabolic enzymes. Indeed, consistent with the metabolite profiling, the expression of the glycolytic components such as the glucose transporter GLUT1, hexokinase 2(HK2) and lactate dehydrogenase A(LDHA) was increased, while the expression of mitochondrial pyruvate carrier (MPC1 and MPC2) were decreased upon *PDHA1* gene inactivation (Figure 3A). In addition, the expression of HIF1α (hypoxia-inducible factor 1) was induced in the *PDHA1* KO cells (Figure 3A).

**Figure 3:** The results of western blotting and RT-PCR assay **A.** shows Western blotting results, where the PDHA1 protein expression in the parental LNCaP cells is strongly positive, but its expression in the *PDHA1* KO cells is almost negative with two different PDHA1 antibodies. Comparatively, the protein expression of the MPC1 and MPC2 is comparatively decreased and the protein expression of the GLUT1, HK2, LDHA, HIF1α, GLS1 and GLUD1 is increased in the LNCaP *PDHA1* KO cells. GAPDH was added as a loading control. **B.** shows the RT-PCR results of the mRNA expression of GLUD1 and GLS1, where the expression of the GLUD1 and GLS1 is significantly increased in the *PDHA1* KO cells, with *P* values of 0.000 and 0.001, respectively, compared to the parental LNCaP cells. **P < 0.01, ***P<0.001.

The article "PDHA1 gene knockout in prostate cancer cells results in metabolic reprogramming towards greater glutamine dependence" was retracted in 2025. Reasons: manipulated images; an official misconduct investigation; duplicated images; overlap with earlier publications.

Considering the profound change of glutamine metabolism pathway in the *PDHA1* KO cells indicated by metabolomic analyses, the glutaminolytic enzymes were investigated firstly by real-time quantitative RT-PCR. There was an increasing expression of the key enzymes GLS1 and GLUD1 in the *PDHA1* KO cells (Figure 3B), indicating activated glutaminolysis. Consistent with the results of the PCR, *PDHA1* KO cells also showed increased expression of the two key enzymes of the glutamine metabolism, GLS1 and GLUD1 at the protein level (Figure 3A). This observation suggested a potential metabolic flux from glutamine to glutamate and then to αKG for the high rate of glutamine catabolism in the *PDHA1* KO cells.

### Glutamine utilization maintains survival and compensates for PDHA1 function loss in prostate cancer cells

As shown in Figure 4A, the PDHA1 KO cells grew more slowly in the RPMI 1640 with 4.0mM L-glutamine compared to the parental LNCaP cells. In order to further determine whether glutamine affected the growth of the human prostate cancer cells with defected *PDHA1* gene, both the parental and *PDHA1* KO cells were cultured with the RPMI 1640 medium without L-glutamine. Cell growth by MTT assay showed significant growth inhibition in the *PDHA1* KO cells without glutamine, although a slight inhibition of cell growth for the parental LNCaP cells was also seen within a period of 7 days' observation (Figure 4A, left panel). The growth inhibition rate due to glutamine deprivation was significantly higher for the PDHA1 KO cells compared to the parental LNCaP cells (Figure 4A, right panel). When such cells were examined with the colony formation assay, there was increasing number of colonies discovered in the parental LNCaP cells with 4mM glutamine in the medium, compared with the parental LNCaP cells in medium without glutamine, even though there was no significant difference between the two groups (*P*=0.760). However, the *PDHA1* KO cells cultivated in the medium with 4mM glutamine demonstrated significantly higher colonies compared to the *PDHA1* KO cells cultivated in medium without glutamine (*P*=0.006), additional evidence of survival and growth reliability of glutamine in the *PDHA1* KO cells (Figure 4B).

The article "PDHA1 gene knockout in prostate cancer cells results in metabolic reprogramming towards greater glutamine dependence" was retracted in 2025. Reasons: manipulated images; an official misconduct investigation; duplicated images; overlap with earlier publications.

**Figure 4:** Effect of glutamine on cell growth, apoptosis, ATP and ROS production **A.** shows the growth inhibition due to glutamine deprivation was significantly higher for the *PDHA1* KO cells compared to the parental cells, especially at day5 (*P=0.001*), day6 (*P<0.001*) and day7 (*P<0.001*). The bars on each detection point represent standard deviations from three independent experiments. **B.** shows the *PDHA1* KO cells cultured in the medium with glutamine form significantly more clones (*P*=0.006) compared to the cells cultured without glutamine, while the parental cells cultured with glutamine shows no significant difference compared to the cells cultured without glutamine (*P*=0.760). **C.** shows strong glutamine addiction of the *PDHA1* KO cells for survival. The *PDHA1* KO cells with glutamine depletion exhibit significantly higher apoptosis rate compared to the cells with 4.0mM glutamine (*P<0.001*) and 5mM dimethyl supplement (*P<0.001*), while no significant apoptosis rate is observed between the parental cells cultured without glutamine and neither with glutamine (*P*=0.094) nor 5mM dimethyl αKG (*P*=0.059). **D.** Glutamine addition in the medium recovers the ATP production in the *PDHA1* KO cells. When the cells were cultivated in the medium without glutamine, there are 5.1193 and 3.0758nmol ATP/mg protein in the parental and *PDHA1* KO cells, respectively (*P*<0.001). However, when both of the cells were cultivated in the medium with glutamine, 5.4200 and 4.9408nmol ATP/mg protein could be observed (*P*=0.217) in the parental and *PDHA1* KO cells, respectively. The measured ATP concentration was normalized by total protein concentration in each sample. The data are presented as means ± S.D (n=5). **E.** Glutamine addition in the medium decreased the ROS production in the *PDHA1* KO cells. Left panel is the representative images of DCFH flow cytometry of each group. The right panel is the relative mean DCFH fluorescence intensities presented as percentage relative to the control value. There are significantly less ROS detected in the *PDHA1* KO cells cultured in medium with glutamine compared to the cells cultured in the medium with glutamine depletion (*P*=0.016), while there is no significant difference of ROS detection for the parental cells cultured in medium with or without glutamine (*P*=0.443). The data are expressed as mean ± S.D. of 3 independent experiments. *P < 0.05, **P < 0.01, ***P<0.001, according to the 2-tailed Student's t test.

To be sure of the glutamine dependence, we exposed the cells to media with and without glutamine and measured its ability to prevent apoptosis. It was repeatedly verified that glutamine removal significantly induced apoptosis in both the parental and *PDHA1* KO cells (Figure 4C). Because it was indicated that glutamine feeds the TCA cycle in many cancers [10, 11], we hypothesized that glutamine removal-induced apoptosis might result from the TCA cycle inhibition. To verify this possibility, we replaced glutamine with a cell penetrable form of αKG (dimethyl α-ketoglutarate) in the medium in order to investigate whether dimethyl αKG could improve the cell survival. It was observed that the TCA cycle intermediate αKG prevented glutamine removal-induced apoptosis in both cell types, but the effect was only significant in the *PDHA1* KO cells (Figure 4C), a result implying that these *PDHA1* KO cells were more vulnerable in medium without the αKG precursor glutamine.

The article "PDHA1 gene knockout in prostate cancer cells results in metabolic reprogramming towards greater glutamine dependence" was retracted in 2025. Reasons: manipulated images; an official misconduct investigation; duplicated images; overlap with earlier publications.

To determine the effects of glutamine on energy homeostasis in prostate cancer cells, the cells were cultured with various concentrations of glutamine for 24hrs, and the effect of glutamine on ATP production was monitored. Our data showed that ATP level of *PDHA1* KO cells was significantly lower (*P*<0.001) than that of the parental cells, and such low level of ATP could be mostly alleviated by 4mM glutamine treatment (Figure 4D; *P*=0.217), suggesting that glutamine could partly improve cellular ATP production in the PDHA1 KO prostate cancer cells.

To reveal the effect of glutamine on intracellular ROS generation, DCFH-DA assay was performed (Figure 4E). The level of intracellular ROS was significantly higher in the LNCaP *PDHA1* KO cells compared to the parental LNCaP cells (*P*=0.016) in the medium without glutamine. Intracellular ROS levels in both types of cells decreased upon glutamine treatment, and this effect was only prominent in the KO cells.

### PDHA1 knockout cells are more vulnerable to glutaminase and glutamate dehydrogenase inhibitors

Since *PDHA1* KO cells demonstrated increased sensitivity to glutamine deprivation, we used glutaminase inhibitors bis-2-(5 phenylacetamido-1, 2, 4-thiadiazol-2-yl) ethyl sulfie (BPTES) and epigallocatechin-3-gallate (EGCG) to treat both cell lines, in order to explore the effect of glutaminolysis pathway on the *PDHA1* KO cell survival. Firstly, the morphology of the cells treated with different concentrations of BPTES and EGCG was analyzed (Figure 5A). When the parental LNCaP cells were treated with these inhibitors for 48hrs, the cell number was decreased and there were a number of floating cells in the medium (Figure 5A, upper panel). But, when the *PDHA1* KO cells were treated with the same inhibitors with the same concentrations, there were apparently fewer living cells and more floating cells observed, compared to the cells treated with DMSO or PBS as controls (Figure 5A, lower panel).

The article "PDHA1 gene knockout in prostate cancer cells results in metabolic reprogramming towards greater glutamine dependence" was retracted in 2025. Reasons: manipulated images; an official misconduct investigation; duplicated images; overlap with earlier publications.

**Figure 5:** The glutaminase inhibitor BPTES and glutamate dehydrogenase inhibitor EGCG impair cell survival in the PDHA1 KO cells **A.** shows represent morphology of the cells treated with control, BPTES and EGCG of indicated concentrations for 48hrs. The scale bar is 100μm. **B.** BPTES significantly induces apoptosis in the parental and *PDHA1* KO cells. Cell survival and apoptosis were assessed by flow cytometry analysis of Annexin-V binding. **C.** EGCG induces greater apoptosis in the *PDHA1* KO cells. Cell survival and apoptosis was assessed by flow cytometry analysis of Annexin-V binding. **D.** BPTES and EGCG increase the ROS in the *PDHA1* KO cells. Left panel represents images of DCFH flow cytometry of each group. The right panel is for the relative mean DCFH fluorescence intensities. The data are expressed as the mean ± S.D. of 3 independent experiments. *P < 0.05, **P < 0.01, ***P<0.001, according to 2-tailed Student's t test.

Then the effect of the inhibitors on apoptosis and ROS production was analyzed with flowcytometry. As shown in Figure 5B, 10μM BPTES treatment induced apoptotic cells (*P*=0.212) and 20μM BPTES treatment induced even more apoptotic cells in the parental LNCaP cells (*P*=0.012). However, 10μM BPTES treatment induced significantly more apoptotic cells (*P*=0.005) and 20μM BPTES induced even more apoptotic cells in the PDHA1 knockout cells (*P*=0.000, Figure 5B). Similarly, 25μM EGCG treatment induced apoptotic cells (*P*=0.014) and 50μM EGCG treatment induced even more apoptotic cells in the parental cells (*P*=0.007). Again, 25μM EGCG treatment induced significantly more apoptotic cells (*P*=0.002) and 50μM EGCG induced even more apoptotic cells in the *PDHA1* KO cells (*P*=0.000, Figure 5C). As shown in Figure 5D, applications of 10μM BPTES and 25μM EGCG in both types of cells significantly increased the production of ROS. Collectively, the above results indicated the vulnerability of the *PDHA1* KO cells to the inhibitors.

### Strong GLS1 and GLUD1 protein expression in prostate cancers predicts poor clinical outcome

Immunohistochemically, the positivity of the key enzymes utilized for glutaminolysis, GLS1 and GLUD1 were confined in the cytoplasm of the tumor cells. Variable degrees of immunoreactivity were observed in the prostate cancer samples. Neither pure negative GLS1 nor pure negative GLUD1 protein expression was revealed. To determine the clinical relevance associated with the glutaminolysis, we evaluated the association of individual protein expression levels with the clinical and pathologic characteristics (Table 1). Both of the two protein expression were significantly positively correlated with the Gleason scores (Figure 6A–6F) in the prostate cancers (*P*=0.017 and 0.021, respectively). Kaplan-Meier analysis showed that higher levels of GLUD1 and GLS1 expression were significantly associated with shorter overall survival in univariate test (Figure 6G and 6H, *P*=0.023 and 0.001 respectively). Collectively, these results suggested that high levels of GLUD1 and GLS1 expression were potential prognostic biomarkers for prostate cancer, an attractive target for therapeutic intervention.

The article "PDHA1 gene knockout in prostate cancer cells results in metabolic reprogramming towards greater glutamine dependence" was retracted in 2025. Reasons: manipulated images; an official misconduct investigation; duplicated images; overlap with earlier publications.

**Table 1:** The associations between the expression of GLS1 and GLUD1 in prostate cancers and the clinicopathological characters

	**Total**	**GLS1 expression**		**P value**	**GLUD1 expression**		**P value**
		**Low**	**High**		**Low**	**High**	
Ages				0.114			0.419
<70	45	32(71.1%)	13(28.9%)		21(47.7%)	24(53.3%)	
≥70	42	23(54.8%)	19(45.2%)		16(38.1%)	26(61.9%)	
Gleason score				0.017*			0.021*
<5	45	30(66.7%)	15(33.3%)		21(46.7%)	24(53.3%)	
5-7	23	18(78.3%)	5(21.7%)		13(56.5%)	10(43.5%)	
≥8	19	7(36.8%)	12(63.2%)		3(15.8%)	16(84.2%)	
PSA				0.491			0.648
<100	40	23(57.5%)	17(42.5%)		17(42.5%)	23(57.5%)	
≥100	40	26(65.0%)	14(35.0%)		15(37.5%)	25(62.5%)	
UIGG stage				0.886			0.637
I-II	66	44(63.6%)	24(34.4%)		29(43.9%)	37(56.1%)	
III-IV	21	13(61.9%)	8(38.1%)		8(38.1%)	13(61.9%)	

* *P* < 0.05, **P < 0.01, ***P<0.001

**Figure 6:** GLS1 and GLUD1 are over-expressed in prostate cancers and associated with poor survival Immunohistochemical staining of GLS1 in human prostate cancers with Gleason score 4 **A.**, 7 **B.** and 9 **C.** Immunohistochemical staining of GLUD1 in human prostate cancers with Gleason score 4 **D.**, 7 **E.** and 9 **F.** **G.** Kaplan-Meier survival curves of the 87 patients with prostate cancer expressing high (blue-line) or low (green-line) GLS1 protein. **H.** Kaplan-Meier survival curves of the 87 patients with prostate cancer expressing high (blue-line) or low (green-line) GLUD1 protein. Log-rank *P* value is shown. The scale bar in the Figure 6 3A to F is 100μm.

## DISCUSSION

In this study, we reported that prostate cancer cells developed alternative metabolic compensatory strategies for survival and growth when their energy metabolism was forced to change *in vitro*. Our study demonstrated that the suppression of glucose into the TCA cycle through the *PDHA1* KO resulted in rewiring toward enhanced glutamine metabolism by increasing GLS1 and GLUD1 expression, leading to glutamine-dependent cell survival. In addition, the *PDHA1* KO cells grew more slowly compared to the parental LNCaP prostate cancer cells. Although the exact mechanism behind this is currently not fully clear, it is most probably due to the dysfunctional mitochondria created by the mitochondrial gate-keeper gene *PDHA1* knockout, which resulted in abnormal ROS and ATP productions in the cells. We also showed that targeting the glutaminolysis in the *PDHA1* KO cells could significantly impair the cell growth by inducing apoptosis. These findings pointed to a selective role for GLS1 and GLUD1 in cancer cells, which were prone to utilize glutamine to provide a carbon source for oxidative phosphorylation and to maintain redox balance required for cellular proliferation. Furthermore, strong GLS1 and GLUD1 expression predicted poor clinical outcome in prostate cancers. These results revealed that glutamine utilization, underscoring the flexibility of cellular metabolism, could be a promising target in the prostate cancer.

The article "PDHA1 gene knockout in prostate cancer cells results in metabolic reprogramming towards greater glutamine dependence" was retracted in 2025. Reasons: manipulated images; an official misconduct investigation; duplicated images; overlap with earlier publications.

Cancer cells take up and metabolize glucose and glutamine to a degree that far exceeds their needs for these molecules in anabolic macromolecular synthesis [21, 22]. The mitochondrial PDH plays a crucial role in regulation of glucose homoeostasis in mammalian cells. Cancer cells frequently exhibit increased expression of the PDH kinase PDK1, which phosphorylates and inactivates PDH [8, 23]. PDH is the most important enzyme and transforms pyruvate into acetyl-CoA, which, along with the acetyl-CoA from the fatty acid β-oxidation, enters the Krebs cycle to produce ATP and electron donors, including NADH [24]. Increasing evidence indicates that lower level of PDH activity is significantly associated with tumor cells' aerobic glycolysis and malignancies of tumor cells [20, 25].

Considering the crucial role of *PDHA1* in glucose metabolism and low activity in the tumor cells, it was hypothesized that *PDHA1* functional loss leads to the diversion of glucose-derived pyruvate away from mitochondria and is converted to lactate. As a result, *PDHA1* deficient cells might become dependent on glutamine anaplerosis for maintaining the mitochondrial integrity and TCA cycle function. Our current results are largely in line with this hypothesis.

It was reported that glutamine deprivation could induce apoptosis in hepatoma, hybridoma, leukemia, myeloma and fibroblast cells [26–28]. The molecular mechanism may be explained like this: glutamine deprivation stimulates caspase-2, -3 activation and cleaved-PARP expression, and induces cytochrome C to release. In our study, we have shown that glutamine deprivation induces apoptosis in both the parental and *PDHA1* KO LNCaP cells, and the effect is stronger in the *PDHA1* knockout cells. More intriguingly, this effect can be reversed by the αKG, which supporting our hypothesis that activated glutaminolysis/glutamine pathway plays an important compensatory role in the *PDHA1* KO cells.

The article "PDHA1 gene knockout in prostate cancer cells results in metabolic reprogramming towards greater glutamine dependence" was retracted in 2025. Reasons: manipulated images; an official misconduct investigation; duplicated images; overlap with earlier publications.

The ROS production has been associated with the bioenergetic and biosynthetic state of cancer cells [29, 30]. In our study, we show that the *PDHA1* KO cells have more ROS production compared with the parental cells, which may be due to the complex metabolic reprograming changes. The cells may experience a series of intermediate steps involving anaplerotic processes balancing OXPHOS function and antioxidant defense. We found that the *PDHA1* KO cells indeed showed increased ROS production, although the molecular mechanism is not clear yet. The increased ROS should have negative effect on the cell survival. It is known that high ROS can inhibit SIRT1 and activate p53, contributing to apoptosis and senescence [31, 32]. In addition, it is recently demonstrated that high ROS causes mitochondrial disruption, leading to cytochrome C to release and the subsequent activation of a protease cascade [33], culminating in loss of cell integrity, DNA fragmentation and premature exhaustion of self-renewal of these cells [34, 35]. The glutamine, in addition to supplying anaplerotic carbon for entry into the TCA cycle, played a significant role in maintenance of redox homeostasis. Glutamine is involved in antioxidant defense function in cells by increasing glutathione (GSH) levels, a key component in the body's scavenging defense mechanism against oxidative stress, decreasing ROS levels and providing a source of NADPH, which in turn protected cells from oxidative stress [36]. A recent study showed that glutamine deprivation significantly inhibited self-renewal, decreased expression of stemness related genes, increased intracellular ROS, and induced apoptosis in pancreatic ductal adenocarcinoma (PDAC) cells. The glutamine deprivation significantly increased radiation-induced ROS and sensitized pancreatic cancer stem cells to fractionated radiation [37]. It was also reported that the mitochondrial glutaminolysis contributed to redox homeostasis in cancer cells by mitochondrial enzyme GLUD1, which is commonly upregulated in human cancers. GLUD1 is important for redox homeostasis in cancer cells by controlling the intracellular levels of its product αKG and subsequent metabolite fumarate. Mechanistically, the fumarate can bind to and activate a reactive oxygen species scavenging enzyme glutathione peroxidase 1 to keep redox homeostasis in balance and then maintain cancer cell proliferation and tumor growth [38]. In our present study, we have demonstrated glutamine supplementation in the *PDHA1* KO cells can scavenge the ROS, elevate the Mt ΔΨ(data not shown) and generate ATP. Collectively, our current study confirmed that the *PDHA1* KO prostate cancer cells were more dependent on glutamine anaplerosis for survival.

The article "PDHA1 gene knockout in prostate cancer cells results in metabolic reprogramming towards greater glutamine dependence" was retracted in 2025. Reasons: manipulated images; an official misconduct investigation; duplicated images; overlap with earlier publications.

Inhibition of mitochondrial pyruvate metabolism might increase glutamate-dependent anaplerosis and promote reductive metabolism of αKG to supply citrate for lipid synthesis [39]. It has been shown that under glucose deprivation, glutamine-derived fumarate, malate, and citrate contribute to the survival and proliferation in tumor cells [10]. In our present study, we have shown that *PDHA1* KO prostate cancer cells become even more dependent on glutaminolysis to supply cellular ATP and scavenge ROS production. Glutamine actively participated in the alternative energy metabolism and antioxidant defense of cancer cells when such cancer cells were forced to obtain energy through glycolysis, in order to maintain cell growth and survival in the *PDHA1* KO prostate cancer cells.

Our results also showed that GLS1 and GLUD1 were differentially expressed at the cytoplasm of prostate cancer cells (Figure 6A-F) and patients with tumors harboring high expression of GLS1 and GLUD1 had a significantly lower survival rate than those patients with tumors of low GLS1 and GLUD1 expression (Figure 6G and 6H). Targeting glutamine metabolism had recently emerged as a promising approach in cancer treatment, as it affected the energy generation, survival, and growth of cancer cells [40]. Recognition of the role of glutamine metabolic pathway as an alternative source of energy and anabolic building block offered one of the most promising targets for anticancer strategies [41]. It is reported that targeting glutaminolysis has anti-leukemic activity in acute myeloid leukemia and synergizes with BCL-2 inhibition [42]. The glutamine addicted melanoma cell lines, could be treated with aminooxyacetate or glutamine depletion [43].

Another recent report also showed that *MYCN*-amplified neuroblastoma cells predominantly rely on activation of ASCT2 to maintain sufficient levels of glutamine essential for TCA cycle anaplerosis and biosynthetic and the ASCT2 activation coordinate to ATF4 and N-Myc might contribute to aggressive neuroblastoma progression [44]. Similarly, glutamine deprivation enhanced antitumor activity of 3-bromopyruvate through the stabilization of monocarboxylate transporter-1 [45]. All of these studies supported the notion that targeting glutamine metabolism is a promising therapeutic approach synergizing with other anticancer regents. Thus, intervention in the glutamine metabolic processes may provide novel approaches to improve cancer treatment. For example, the development of small molecule inhibitors to effectively inhibit glutaminolytic enzymes including GLS and GLUD can both increase cancer cell susceptibility to apoptosis and undo tumorigenic metabolic reprogramming, providing better therapeutic modality in cancer treatment [46].

The article "PDHA1 gene knockout in prostate cancer cells results in metabolic reprogramming towards greater glutamine dependence" was retracted in 2025. Reasons: manipulated images; an official misconduct investigation; duplicated images; overlap with earlier publications.

In summary, our data have demonstrated forced deficiency of *PDHA1* expression by KO in prostate cancer cells results in metabolic reprogramming towards higher glutaminolysis, a process being preferentially vulnerable to glutamine inhibitors. Further clinical sample analyses have revealed higher levels of the glutaminolysis-related genes expression, including GLUD1 and GLS1, and positive GLUD1 and GLS1 protein expression are significantly associated with shorter clinical outcome in the prostate cancers. Collectively, our current results highlight the importance of targeting glutaminolysis as a promising therapeutic option for prostate cancer.

## MATERIALS AND METHODS

### Cell lines and reagents

The prostatic cancer cell line LNCaP was obtained from ATCC (American Type culture collection, USA) and maintained in our laboratory for the study. Cells were cultured in RPMI 1640 (Gibco™, 32404-014), supplemented with 10% fetal bovine serum (Gibco™, 10500-064) with or without 4mM L-glutamine (Gibco™, 25030-081), 100 U/ml of penicillin and 100ug/ml streptomycin (15140122, Life Technologies) at 37°C, and 5% CO2. Anti-PDH antibody (cell signaling, C54G1), anti-Pyruvate Dehydrogenase E1-alpha subunit antibody (ab110334), monoclonal anti-GAPDH antibody (sigma, AB2302), anti-GLUT1 antibody (cell signaling, D3J3A), Anti-LDHA antibody (abcam, ab47010), anti-HK2 (abcam, ab104836), anti-GLS1 (sigma, WH0002744M1-100UG), anti-GLUD1 (Novus Biologicals, NBP1-54961), anti-MPC1 (Novus Biologicals, NBP1-91706) and anti-MPC2(abcam, ab111380) were applied in the current study. BPTES (SML0601), EGCG (03970590-10MG) and dimethyl-αKG (34963-1) were obtained from Sigma-Aldrich (Sigma-Aldrich Norway AS Oslo, Norway). Annexin-V was purchased from Life technologies (Life technologies, A13199).

### Generation of stable PDHA1 KO cell line

72hrs after the cells were transected with specific TALEN-PDHA1 plasmids, the cells were harvested to prepare single cell suspension of 1cell/100μl by using limiting dilution assay. In short, 100ul/well cell suspension was placed in 96-well plate for culture for 1-3 weeks. Cells from single clones were collected and diluted to 1cell/100μl and cultured in new 96-well plate again. Monoclonal cells were obtained after two rounds of such screening. Genome DNA of the monoclonal cells was prepared for specific *PDHA1* DNA PCR amplification using the primer (Table 2) flanking potential *PDHA1* mutation area and such DNA was applied for sequencing, in order to verify the KO status. The knockout effect of the TALEN constructs was further evaluated by the Western blotting of PDHA1 protein. A separate manuscript for detailed procedure of the *PDHA1* KO LNCaP cell line establishment was submitted.

The article "PDHA1 gene knockout in prostate cancer cells results in metabolic reprogramming towards greater glutamine dependence" was retracted in 2025. Reasons: manipulated images; an official misconduct investigation; duplicated images; overlap with earlier publications.

**Table 2:** The primer sequences applied in the study

**Primers**	**Forward**	**Reverse**
*PDHA1*	TCTGGCGCTGATACCCAATG	CCTCTTGAGCACACCGACTT
*GLS1*	TCCCCAAGGACAGGTGGAA	GAGGTGTGTACTGGACTTGGT
*GLUD1*	TGCATGGCTTAACCTGGTGAT	TCTGGGCAGCTCACAATAAAGT
*β-actin*	CGTCACCAACTGGGACGACA	GGGGTGTTGAAGGTCTCAAA

### Clinical samples of prostate carcinomas

A total of 87 prostate cancer samples were collected from the file of Department of Pathology, the First Affiliated Hospital of Zhengzhou University. The current project using the clinical samples was approved by the First Affiliated Hospital of Zhengzhou University medical ethics committee. All patients provided written informed consent. All the tumors were histologically classified based on the Gleason system and all the classification was re-evaluated by two pathologists.

### Immunohistochemistry(IHC) analysis

The IHC was performed using the EnvisionTM+System. Shortly, sections were deparaffinized by PT-Link machine for 1 hour and 20 minutes and blocked with peroxidase blocking (Dako) for 5 minutes after rinsing by DAKO wash buffer. Then the slides were incubated with the primary antibody at 4°C overnight followed with mouse or rabbit linker for 15 minutes and HRP for 30 minutes at room temperature. The slides were then stained with 3,3′-diaminobenzidine tetrahydrochloride (DAB, Dako) for 5 minutes, counter-stained with hematoxylin, dehydrated and mounted in Richard-Allan Scientific Cytoseal XYL (Thermo Scientific, Waltham, MA, USA). The corresponding non-immune rabbit IgG and non-immune mouse IgG were used as negative controls for GLUD1 and GLS1, respectively.

### Evaluation of IHC staining

Both of the intensity and the extent of immunological staining were analyzed semi-quantitatively. Sections with no labeling or fewer than 5% labeled cells were scored as 0. 15–25%, 25–50%, and more than 50% labeled cells were scored as 1, 2 and 3 respectively. The staining intensity was scored similarly, with 0 used for negative staining, 1 for weakly positive, 2 for moderately positive and 3 for strongly positive. The scores for the percentage of positive cells and the staining intensity were multiplied to generate an immune-reactive score for each specimen, and the scores were finalized and graded as followings: 0 was graded as no expression, 1-4 was graded as low expression and 6-9 was graded as high expression. Each sample was examined separately and scored by two pathologists. The photos were prepared with a Leica DMLB light microscope equipped with SPOT Advanced Software (Olympus, Nagano, Japan).

The article "PDHA1 gene knockout in prostate cancer cells results in metabolic reprogramming towards greater glutamine dependence" was retracted in 2025. Reasons: manipulated images; an official misconduct investigation; duplicated images; overlap with earlier publications.

### Western blotting

For the analysis of protein expression, cells were lysed in RIPA buffer containing a cocktail of protease inhibitors. Lysates were transferred in Eppendorf tubes and centrifuged at 12 000 g for 10 minutes at 4°C before aliquots of 35μg proteins were mixed with loading buffer at 4°C, warmed at 95°C for 5 min and loaded on a 10% gel for SDS-PAGE. After electrophoresis, the proteins were transferred to polyvinylidene difluoride transfer membrane(PVDF) in a Trans-blot apparatus(Bio-Rad, Hercules, CA). Membranes were blocked in 5% milk (Bio-Rad, Hercules, CA) and incubated with the indicated antibodies. After washing with TBST (TBS with 0.1% Tween), corresponding secondary antibodies conjugated with horseradish peroxidase-conjugated (HRP) were then used to incubate the membranes. The samples were finally treated with enhanced chemilluminescence assay reagents (GE Healthcare) and exposed to X-ray film to detect the protein bands. The band intensity was normalized to GAPDH analyzed using Image Lab 2.0 Software (Bio-Rad Laboratories Inc, USA).

### Quantitative real-time polymerase chain reaction (PCR)

Total RNA was extracted from cells using an RNease Mini Kit (Qiagen, Hilden, Germany) and each RNA sample (3μg) was subjected to cDNA synthesis by means of RNA transcription kit (Thermo Fisher scientific, America). Quantitative real-time PCR was performed using the Quantitative SYBR Green PCR Kit (Thermo Fisher scientific, America) on the ABI PRISM 7500 Fast system (Applied Biosystems, Life Technologies, America). All experiments were performed as specified in the manufacturer's protocols. The primers used are shown in Table 2. All samples were analyzed for 3 parallel samples and repeated at least 3 times, and the relative expression of the target gene was calculated with 2^−ΔΔCt^ values with the Application Relative Quantification Study Program (Applied Biosystems, Life Technologies, America).

### Cell proliferation assay

Cells from the prostate cancer cell line LNCaP and the LNCaP-PDHA1 knockout cell line were seeded at 500cells/well in 96-well plates in RIMP1640 media and cultured for 24 hrs. Then the culture media were removed and replaced with new media with different concentrations of glutamine for continuing culture for up to 7 days before the cells were applied in different time intervals for MTT measurements. Cell proliferation was measured by adding 20μl MTT solution (5mg/ml) per well for an additional incubation of 4 hrs. The MTT reaction was terminated through the replacement of the medium by 200μl of DMSO. The absorbance at 490nm was measured using a microplate reader (Biochrom Asys UVM340, Biochrom Ltd ). Each experiment was performed in triplicate and repeated three times to assess for consistency of results.

The article "PDHA1 gene knockout in prostate cancer cells results in metabolic reprogramming towards greater glutamine dependence" was retracted in 2025. Reasons: manipulated images; an official misconduct investigation; duplicated images; overlap with earlier publications.

### Annexin-V assay

The effect of glutamine deprivation and glutaminolysis inhibition on cell apoptosis was detected by using Annexin-V FITC Kit. Briefly, 1.7×10^5^ cells/well were seeded into the six-well plates overnight, and then the cells were cultured in the media with 10 and 20μM BPTES or 25 and 50μM EGCG with or without glutamine for 48 hrs. The cells were detached by 0.25% Trypsin without EDTA before collected. After PBS washing, the cells were resuspended in 500μl Annexin-V and PI dual-stain solution (0.1mg of Annexin-V FITC and 1 mg of PI) for 15min in dark and detected by BD LSR II flow cytometer (BD Biosciences). FCS4 Express Software was applied for further analyses of the flowcytometry results. Each experiment was repeated at least twice for consistency of response.

### Glucose consumption assay

The glucose consumption was determined by a glucose assay kit (Glucose Determination kit GAHK-20, Sigma-Aldrich) according to the manufacturer's instruction. In brief, the cells were seeded in 6 well plates at 5×10^5^ cells/well/2ml in the corresponding culture medium for 12 and 24hrs, and then the media were removed and the concentration of glucose in the medium was measured using a Biochrom Assays UVM340 Microplate Reader. The glucose consumption was calculated by the original medium concentration minus the glucose concentration in the medium after 12 or 24hrs. Data were normalized based on the viable cell counts measured by the MTT assays. All the experiments were performed in triplicate and repeated twice.

### Measurement of L-glutamine level

Briefly, cells were plated at 1×10^5^ cells per well in 24-well culture plates (Costar) and allowed to adhere overnight. After 24 and 48hrs the cell culture media were collected and centrifugated at 10,000 × g for 5min. at 4°C. 1-40μl of the supernatant were collected and added into desired well(s) in a 96-well plate. The L-glutamate level in the media was measured following the manufacturer's instructions (Glutamine Colorimetric Assay Kit, K556-100), and the L-glutamine consumption was calculated by the original medium concentration minus the L-glutamate concentration in the medium detected.

### ATP assay

Cellular ATP production was assessed by using Luminometric ATP Assay Kit (ATP determination kit, A22066, life technologies). In short, after the cells were treated with different concentrations of L-glutamine for 24hrs, 90μl/well of the ATP reaction mix was added into the sample and mixed gently before incubated for 10-20 min in dark at room temperature. The luminescence intensity was monitored with a plate reader of Tecan Infinite™ F500, Bioluminescence Resonance Energy Transfer. The ATP levels were normalized based on the viable cell counts measured by the Trypan blue assays. Each experiment was performed in triplicate and repeated twice to assess for consistency of results.

The article "PDHA1 gene knockout in prostate cancer cells results in metabolic reprogramming towards greater glutamine dependence" was retracted in 2025. Reasons: manipulated images; an official misconduct investigation; duplicated images; overlap with earlier publications.

### ROS assay

Intracellular ROS production was detected using 2′,7′-dichlorodihydrofluorescein diacetate (DCFH-DA; Molecular Probes) at a final concentration of 5μM according to the manufacturer's protocol. Following treatment, the cells were washed and incubated with DCFH-DA for 20 min at 37°C in the dark. The fluorescence corresponding to the intracellular ROS levels was monitored and analyzed by flow cytometry (BD FACSCalibur flow cytometer, FACS101; BIO-RAD Corporation).

### Gas chromatography/mass spectrometry (GC/MS)

Cells (1×107) with culture media were initially washed in PBS. The cells were dissolved in 2mL of methanol: water (1:1, v/v) solvent and then scraped off from the culture plastic containers using silicon rubber cell scrapers. The detailed metabolite extraction can be referred to [47]. We investigated the change of metabolites and metabolism pathway using gas chromatography with time-of-flight mass spectrometry (GC/TOFMS)-based metabolomics approach. GC/TOF-MS analysis was performed using an Agilent 7890 gas chromatograph system coupled with a Pegasus HT time-of-flight mass spectrometer. The system utilized a DB-5MScapillary column coated with 5% diphenyl cross-linked with 95% dimethyl polysiloxane (30m×250μm inner diameter, 0.25μm film thickness; J&W Scientific, Folsom, CA, USA). A 1μL aliquot of the analyte was injected in splitless mode. Helium was used as the carrier gas, the front inlet purge flow was 3mL/min, and the gas flow rate through the column was 20mL/min. The initial temperature was kept at 50°C for 1 min, then raised to 330°C at a rate of 10°C/min, then kept for 5min at 330°C. The injection, transfer line and ion source temperature were 280, 280, and 220°C, respectively. The energy was -70eV in electron impact mode. The mass spectrometry data were acquired in full-scan mode with the m/z range of 85-600 at a rate of 20 spectra per second after a solvent delay of 366s. Chroma TOF 4.3X software of LECO Corporation and LECO-Fiehn Rtx5 database were used for raw peaks extracting, the data baselines filtering and calibration of the baseline, peak alignment, deconvolution analysis, peak identification and integration of the peak area [48]. The RI (retention time index) method was used in the peak identification, and the RI tolerance was 5000. Then the Simca-P 12.0.1 software (Umetrics, Umea˚, Sweden) was used for further statistical analysis PCA and OPLS-DA were performed to discriminate between PDHA1 gene KO and the control groups. Those variables with VIP>1.0 were considered relevant for group discrimination. After the multivariate approaches, the significance of each metabolite in-group discrimination was further measured by the Student's t-test (*P*<0.05). A list was obtained with all the metabolites that had important contribution to the variance. Metabolite identification from these selected variables was subsequently achieved by NIST 05 Standard mass spectral databases (NIST, Gaithersburg, MD) and available reference standards, separately. Metabolic pathway analysis was then performed via MetaboAnalyst 2.0 to identify the affected metabolic pathways analysis and visualization.

The article "PDHA1 gene knockout in prostate cancer cells results in metabolic reprogramming towards greater glutamine dependence" was retracted in 2025. Reasons: manipulated images; an official misconduct investigation; duplicated images; overlap with earlier publications.

### Statistics

Results for the GC-MS are shown as mean ± standard error of the mean (SEM). PCA was performed using commercially available SIMCA-P Plus Software, version 12.0.1 (Umetrics). Tukey-Kramer honest significance testing was performed for multiple comparison testing. SPSS software (version 18.0) was used for other data analyses. Values are shown as mean ± standard deviation (SD) or SEM. Data were analyzed using the Student's t test or one-way ANOVA. Survival analysis was performed using the Kaplan-Meier method, and groups were compared with log-rank tests. Patients alive on the last follow-up date without recurrence were censored. For all the analyses, associations were considered to be significant if the *P* value<0.05.
